The article "Bioactive Fraction of Annona reticulata Bark (or) Ziziphus jujuba Root Bark along with Insulin Attenuates Painful Diabetic Neuropathy through Inhibiting NF-κB Inflammatory Cascade" was published in 2017. Journal: Front Cell Neurosci.

# Bioactive Fraction of *Annona reticulata* Bark (or) *Ziziphus jujuba* Root Bark along with Insulin Attenuates Painful Diabetic Neuropathy through Inhibiting NF-κB Inflammatory Cascade

**DOI:** 10.3389/fncel.2017.00073

**Published:** 2017-03-22

**Authors:** Raghuram Kandimalla, Suvakanta Dash, Sanjeeb Kalita, Bhaswati Choudhury, Sandeep Malampati, Rajlakshmi Devi, Muthiah Ramanathan, Narayan C. Talukdar, Jibon Kotoky

**Affiliations:** ^1^Drug Discovery Laboratory, Institute of Advanced Study in Science and TechnologyGuwahati, India; ^2^Girijananda Chowdhury Institute of Pharmaceutical ScienceGuwahati, India; ^3^School of Chinese Medicine, Hong Kong Baptist UniversityKowloon Tong, Hong Kong; ^4^PSG College of PharmacyCoimbatore, India; ^5^National Institute of Pharmaceutical Education and ResearchGuwahati, India

**Keywords:** neuro-inflammation, diabetic neuropathic pain, NF-κB, iNOS, cytokines, oxidative stress

## Abstract

The present study explains the neuroprotective ability of bioactive fractions of *Annona reticulata* bark (ARB) and *Ziziphus jujuba* root bark (ZJ) along with insulin against diabetic neuropathy. By using different solvents of increasing polarity ARB and ZJ were undergone for bioactive guided fractionation. The neuroprotective ability of the all the plant fractions were tested against H_2_O_2_ induced toxicity in SHSY5Y neuroblastoma cell lines and DRG neuronal cells. Among all the fractions tested, the methanol extract of ARB and ZJ (ARBME and ZJME) and its water fractions (ARBWF and ZJWF) exhibited significant neuroprotection against H_2_O_2_ induced toxicity in SHSY5Y cells and DRG neuronal cells. Further both the active fractions were tested against streptozotocin (55 mg/kg i.p.) induced diabetic neuropathy in male Wistar rats. Body weight changes, blood glucose levels and pain threshold through hot plate, tail immersion, cold plate and Randall-Sillitto methods were measured throughout the study at weekly interval. After completion of the drug treatment period, all the animals were sacrificed to measure the sciatic nerve lipid peroxidation, antioxidative enzyme levels (SOD, catalase, and GSH) and cytokine levels (IL-1β, IL-6, IL-10, TNF-α, iNOS, and NFκB) through ELISA and western blotting analysis. Results of this study explain that ARBME, ZJME, ARBWF, and ZJWF along with insulin potentially attenuate the thermal, mechanical hyperalgesia and cold allodynia in diabetic neuropathic rats, where insulin treatment alone failed to diminish the same. Reduction of sciatic nerve oxidative stress, NF-κB and iNOS mediated inflammatory cascade and normalization of abnormal cytokine release confirms the possible mechanism of action. The present study confirms the neuroprotective ability of ARB and ZJ against painful diabetic neuropathy through inhibiting oxidative stress and NF-κB inflammatory cascade.

The article "Bioactive Fraction of Annona reticulata Bark (or) Ziziphus jujuba Root Bark along with Insulin Attenuates Painful Diabetic Neuropathy through Inhibiting NF-κB Inflammatory Cascade" was published in 2017. Journal: Front Cell Neurosci.

## Introduction

According to the World Health Organization (WHO) report by 2014, 422 million world populations are suffering from diabetes, which gives the status of an epidemic around the globe. Prolonged or untreated diabetic patients suffer from a chronic condition called neuropathy which diminishes the quality life of wellbeing. Around 20–24% of diabetic patients suffer from diabetic neuropathy (DN). Pain is the main symptom of DN, which is characterized by thermal, mechanical hyperalgesia and cold allodynia. The mechanism behind precipitation of diabetic neuropathic pain (DNP) is still unclear (Dyck et al., 2000; Kaeidi et al., 2011; Kandhare et al., 2012). Hyperglycemia and its associated metabolic disarrangements are the primary cause of deterioration of neurons and DNP. The experimental and clinical evidences concluded that long term hyperglycemic condition mediated cellular dysfunctions plays a pivotal role in nerve injury through oxidative stress, cytokine release and neuro-inflammation. Increased blood glucose level also causes the activation of polyol pathway and advanced glycation end products (AGEs) which in turn stimulates the NF-κB inflammatory cascade and releases the oxidants (Yagihashi et al., 2011; Babizhayev et al., 2015).

Reports suggested that treatment with anti-oxidant molecules along with strict hyperglycemic control attenuates the DNP (Yagihashi et al., 2011). Where, strict glycemic control alone through insulin therapy can not diminish the risk (Tiwari et al., 2011). Current drug treatment regimen is incapable to completely relief the DNP, which includes anti-hyperglycemics, sodium and calcium channel blockers, opioids, anti-depressants, anticonvulsants, etc. This complex medication can leads to serious side effects that diminish the quality of life and increases the financial burden on patients. Despite having a large number of drugs in the market still, the management of diabetic complications is a substantial challenge (Honore et al., 2011; Peng et al., 2015). Various reports from preclinical data suggested that herbal extracts from *Curcuma longa, Tribulus terrestris, Emblica officinalis* (Ranjithkumar et al., 2013) have beneficial effects in the management of DNP. In this study, we evaluated the neuroprotective ability of two medicinal plants *Ziziphus jujuba* and *Annona reticulata* against painful DNP. These two plants have been using for curing different diseases like diabetes, inflammation and liver ailments by various tribal communities of northeast India but there is no scientific validation for the same. Bioactive fractions of these two plants (*A. reticulata* and *Z. jujuba)* have the ability to protect the hepatocytes and reduce the inflammation (Kandimalla et al., 2016a,e).

The article "Bioactive Fraction of Annona reticulata Bark (or) Ziziphus jujuba Root Bark along with Insulin Attenuates Painful Diabetic Neuropathy through Inhibiting NF-κB Inflammatory Cascade" was published in 2017. Journal: Front Cell Neurosci.

*Ziziphus jujuba* Mill. (Rhamnaceae) commonly known as Indian date or red date, a spiny shrub to small tree widely available in tropical and warm subtropical regions around the world. This plant is widely used in traditional system of medicine for different ailments like diabetes, inflammation, infections, liver diseases, and throat problems by local tribal peoples in India (Naik et al., 2013). *Z. jujuba* contains phenolic and flavonoid compounds (San and Yildirim, 2010; Wang et al., 2016), polysaccharides (Yue et al., 2014), triterpenoid acids (Guo et al., 2009), alkaloids and glycoside compounds (Meng et al., 2013). Different plant parts of *Z. jujuba* were reported to have antioxidant (Sun et al., 2011), anti-inflammatory (Yu et al., 2012), hepatoprotective, anti-tumor (Hoshyar et al., 2015) and induction of erythropoietin expression (Lam et al., 2016) activities.

*Annona reticulata* L. (AR) is a small tree belongs to the family Annonaceae which is widely available in tropical regions of the world, especially in India, China, America, and West Indies (Rahman et al., 2011). Various reports suggests that AR traditionally used as antiparasitic, antidiarrhoeic, antidysenteric and insecticide (Wele et al., 2008). Different parts of the plant were reported to have anticancer, analgesic, anti-inflammatory, antiulcer, antioxidant, hepatoprotective, and wound healing properties (Jamkhande and Wattamwar, 2015; Kandimalla et al., 2016a). The plant has been reported for different phytochemicals like cycloreticulins A and B, cyclooctapeptides (Wele et al., 2008), acetogenins (Chang et al., 1998), cycloreticulin C, glabrin A, cyclopeptides (Wele et al., 2009).

To treat the DNP condition, single therapeutic agent is not sufficient as the drug has to act on the hyperglycemia, oxidative stress and nerve inflammation simultaneously (Sandireddy et al., 2014). Plants are the source for a vast number of bioactive phytoconstituents which have the potential to treat the disease and related complications together. The present study was aimed to investigate the ability of bioactive guided fractions of *Z. jujuba* root bark and *A. reticulata* bark along with insulin against painful diabetic neuropathy. To achieve the goal initially we evaluated the neuroprotective ability of all the plant extract and fractions against SHSY5Y cell line and isolated Dorsal Root Ganglion (DRG) neurons. Further, the active fractions from the *in vitro* study were screened against STZ induced DNP in rats. Findings of the study will give insight regarding successful translation of multicomponent therapeutic strategy for the treatment of DNP.

The article "Bioactive Fraction of Annona reticulata Bark (or) Ziziphus jujuba Root Bark along with Insulin Attenuates Painful Diabetic Neuropathy through Inhibiting NF-κB Inflammatory Cascade" was published in 2017. Journal: Front Cell Neurosci.

## Materials and methods

### Chemicals

3-(4,5-dimethyl thiazol-2-yl)-5-diphe- nyl tetrazolium bromide (MTT), trypan blue and trypsin were obtained from Sigma-Aldrich Co, St Louis, USA. Cell culture media and fetal bovine serum (FBS) were procured from Invitrogen, Life technologies, USA. TNF-α, IL-1β, IL-6, and IL-10 ELISA kits were obtained from RandD systems. Antibodies and nitrocellulose membrane were purchased from Cell Signaling, USA. Superoxide dismutase (SOD) and catalase (CAT) assay kits were procured from Cayman, USA. Biochemical kits were purchased from Accurex Biomedical Pvt. Ltd, Mumbai. Insulin was procured from Abbott, India LTD. All the other chemicals used in this study were of analytical grade and obtained from Sigma-Aldrich Co, St Louis, USA and Merck, Germany.

### Plant collection, identification, extraction, and bioactive guided fractionation of plant materials

The detailed description for the plant collection, identification, extraction and bioactive guided fractionation of both the plants *Z. jujuba* root bark and *A. reticulata* was previously reported from our research group (Kandimalla et al., 2016a,e). Figure 1 depicts the schematic representation of the bioactive guided fraction.

**Figure 1:** **Schematic representation of bioactive guided fractionation of ***A. reticulata*** bark and ***Z. jujuba*** root bark**. ARBME, *A*. *reticulata* bark methanol extract; ARBHF, *A*. *reticulata* bark hexane fraction; ARBCF, *A. reticulata* bark chloroform fraction; ARBEAF, *A*. *reticulata* bark ethyl acetate fraction; ARBWF, *A*. *reticulata* bark water fraction; ARBMR, *A*. *reticulata* bark methanol residue; ZJME, *Z*. *jujuba* root bark methanol extract; ZJHF, *Z*. *jujuba* root bark hexane fraction; ZJCF, *Z*. *jujuba* root bark chloroform fraction; ZJEAF, *Z*. *jujuba* root bark ethyl acetate fraction; ZJWF, *Z*. *jujuba* root bark water fraction; ZJMR, *Z*. *jujuba* root bark methanol residue.

### Evaluation of the effect of plant fractions on H_2_O_2_ intoxicated SHSY5Y cell lines and DRG neurons

#### Cell lines and maintenance

The SHSY5Y neuroblastoma cell line was procured from National Center for Cell sciences (NCCS), Pune, Maharashtra, India. The cells were maintained in culture flasks containing DMEM media supplemented with FBS and antibiotic solution (Sigma-Aldrich, USA) in a humidified 5% CO_2_ incubator at 37°C. Every 2 days the culture medium was replaced with new medium.

For isolation of DRG neuron cells, male wistar rats (2 months old) were anesthetized using ketamine and xylazine cocktail (80 and 10 mg/kg) and the neurons were carefully collected from peripheral nerve roots. The neurons were incubated in DMEM supplemented with 1% streptomycin- penicillin (Sigma-Aldrich, USA). Further connective tissues were removed and ganglia were treated with collagenase-IV (0.28 ml in DMEM), and trypsin (25,000 units/ml in DMEM) for 45 min and incubated at 37°C in CO_2_ incubator. The resulting cell suspension was filtered through 74 μm filter and centrifuged at 1,500 g and further proceed for culturing (Naziroglu et al., 2013; De Luca et al., 2015).

The article "Bioactive Fraction of Annona reticulata Bark (or) Ziziphus jujuba Root Bark along with Insulin Attenuates Painful Diabetic Neuropathy through Inhibiting NF-κB Inflammatory Cascade" was published in 2017. Journal: Front Cell Neurosci.

### Neuroprotective ability of *Z. jujuba* and *A. reticulata* fractions

By using the cell viability (MTT) assay the neuroprotective ability of *A. reticulata* methanol extract and its fractions (ARBME, ARBHF, ARBCF, ARBEAF, ARBWF, and ARBMR) and *Z. jujuba* methanol extract and its fractions (ZJME, ZJHF, ZJCF, ZJEAF, ZJWF, and ZJMR) were determined. Briefly, SHSY5Y cells (1 × 10^4^ cells/well) were seeded into 96 well plates and incubated overnight in a CO_2_ incubator at 37°C. The next day morning culture media from the plate was replaced with fresh media. Cells were pretreated with plant fractions at different concentrations (0, 0.5, 5, and 50 μg/ml) and incubated for 12 h before the cells were exposed to 100 μM H_2_O_2_ for next 12 h. After 24 h of the total incubation period, cell viability was evaluated by MTT assay (Kalita et al., 2015; Kalita S. et al., 2016; Kandimalla et al., 2016b). To each well 10 μl of 4 mg/ml MTT solution was added and incubated at 37°C for 2 h. After the incubation period, the MTT solution was removed from the wells and 100 μl of DMSO solution was added to dissolve the formazan crystals. The color intensity was measured at 560 nm using ELISA microplate reader (Thermo Scientific, USA). Cells were exposed to different treatment groups as given below:

**Group-I (control):**

*Normal control:* Cells treated with 100 μl of serum free culture medium for 24 h.

*DMSO control:* Cells treated with 100 μl of serum free culture medium containing DMSO (0.25% v/v) for 24 h.

*A. reticulata fractions Control:* Cells treated with 100 μl of serum free culture medium containing ARBME, ARBHF, ARBCF, ARBEAF, ARBWF, and ARBMR (200 μg/ml) separately for 24 h.

*Z. jujuba fractions control*: Cells treated with 100 μl of serum free culture medium containing ZJME, ZJHF, ZJCF, ZJEAF, ZJWF, and ZJMR (200 μg/ml) separately for 24 h.

**Group-II (H**_2_**O**_2_ **treatment):** Cells treated with 100 μl of serum free culture medium containing 100 μM H_2_O_2_ for 12 h.

**Group-III (*A. reticulata* Fractions Treatment):** Cells treated with 100 μl of serum free culture medium containing ARBME, ARBHF, ARBCF, ARBEAF, ARBWF, and ARBMR (at 50, 100, and 200 μg/ml) separately for 12 h + 100 μM H_2_O_2_ for next 12 h.

The article "Bioactive Fraction of Annona reticulata Bark (or) Ziziphus jujuba Root Bark along with Insulin Attenuates Painful Diabetic Neuropathy through Inhibiting NF-κB Inflammatory Cascade" was published in 2017. Journal: Front Cell Neurosci.

**Group-IV (*Z. jujuba* fractions treatment):** Cells treated with 100 μl of serum free culture medium containing ZJME, ZJHF, ZJCF, ZJEAF, ZJWF, and ZJMR (at 50, 100, and 200 μg/ml) separately for 12 h + 100 μM H_2_O_2_ for next 12 h.

### Measurement of lactate dehydrogenase (LDH) levels and lipid peroxidation

Culture media from the all the treatment groups were collected after the drug treatment period to measure the LDH levels. Briefly, the culture media was centrifuged at 2,000 rpm for 15 min, and the supernatant was collected to measure the LDH levels using Ecoline diagnostic kit as per the instructions provided by the manufacturer. Each sample was performed in triplicate and, the results were expressed in U/L. Cells from the wells were scrapped and transferred to RIPA lysis buffer. The protein concentration was determined by Lowry method and TBARS was estimated by following Ohkawa et al. (1979).

### Neuroprotective ability of active plant fractions against DRG cells

DRG cells were cultured in a poly-D-lysine pre coated 96 well plate at 2 × 10^4^ cells/well and treatments were given as following:

*Normal control:* DRG cells treated with 100 μl of serum free culture medium for 24 h.

*DMSO control:* DRG cells treated with 100 μl of serum free culture medium containing DMSO (0.1% v/v) for 24 h.

*A. reticulata fractions Control:* DRG cells treated with 100 μl of serum free culture medium containing ARBME and ARBWF (200 μg/ml) separately for 24 h.

*Z. jujuba fractions control*: DRG cells treated with 100 μl of serum free culture medium containing ZJME and ZJWF (200 μg/ml) separately for 24 h.

**Group-II (H**_2_**O**_2_ **treatment):** DRG cells treated with 100 μl of serum free culture medium containing 100 μM H_2_O_2_ for 12 h.

**Group-III (*A. reticulata* fractions treatment):** DRG cells treated with 100 μl of serum free culture medium containing ARBME and ARBWF (at 50, 100, and 200 μg/ml) separately for 12 h + 100 μM H_2_O_2_ for next 12 h.

**Group-IV (*Z. jujuba* fractions treatment):** DRG cells treated with 100 μl of serum free culture medium containing ZJME and ZJWF (at 50, 100, and 200 μg/ml) separately for 12 h + 100 μM H_2_O_2_ for next 12 h.

After 24 h of incubation MTT assay was performed to determine the percentage cell viability.

### Acute toxicity studies

OECD (Organization for Economic Co-operation and Development) guidelines to test chemicals were followed to perform the acute oral toxicity studies. Swiss albino mice of either sex (*n* = 5) were selected randomly for this study. Mice were fasted overnight with free access to water before administration of test drugs. A single dose of ARBME, ARBWF, ZJME, and ZJWF at 2,000 mg/kg and same dose along with 5 IU/kg of insulin was administered separately to three animals each. Animals kept under observation for 14 days and the dose was considered as toxic if mortality observed in 2 out of 3 animals. The experiment was repeated to confirm the toxic dose if mortality observed in 1 out of 3 animals. The study was continued with small doses (300, 50, and 5 mg/kg body weight) on finding the dose as toxic again (Choudhury et al., 2016).

The article "Bioactive Fraction of Annona reticulata Bark (or) Ziziphus jujuba Root Bark along with Insulin Attenuates Painful Diabetic Neuropathy through Inhibiting NF-κB Inflammatory Cascade" was published in 2017. Journal: Front Cell Neurosci.

### Animals and induction of diabetes

Adult male Wistar rats weighing 200–220 gm were used to conduct the *in vivo* experiments. Animals were housed four per cage and maintained at 24°C ± 1°C, with a relative humidity of 45–55% and 12:12 h dark/light cycle and had free access to standard pellet diet (Provimi Animal Nutrition Pvt. Ltd., India) and water throughout the experimental period. All experiments were carried out between 09:00 and 17:00 h. The experimental protocol was approved by the Institutional Animal Ethics Committee (IAEC) of IASST, Guwahati (IASST/IAEC/2014-15/751) and performed by following the guidelines of Committee for Control and Supervision of Experimentation on Animals (CPCSEA). Diabetes was induced in overnight fasted animals by single intraperitoneal injection of freshly prepared streptozotocin (STZ) in citrate buffer (pH: 4.5) at 55 mg/kg. Animals injected with citrate buffer alone considered as control animals. Two percent glucose solution (2 ml/kg) fed to all the animals before STZ injection and diabetes confirmed by measuring the fasting blood glucose (FBG) levels after 5 days of injection. Animals had FBG levels more than 250 mg/dl is considered as diabetic and included in the study (Kalita H. et al., 2016). Body weight and FBG levels were measured every week throughout the study.

### Experimental protocol for diabetic neuropathy

From the *in vitro* study results, *A. reticulata* and *Z. jujuba* methanol extracts (ARBME and ZJME) and its water fractions (ARBWF and ZJWF) were selected for *in vivo* assays. These extracts and fractions were administered separately along with insulin to evaluate against DNP. A total of 72 animals were divided into twelve groups (*n* = 6). Animal's response to different analgesic models before STZ injection was recorded and considered as 0th week reading. After STZ induction animals left untreated for 4 weeks to precipitate diabetic neuropathic condition and from the starting of 5th week, drug treatment schedule started as follows:

**Group-I:** Normal animals + vehicle treatment (0.3% carboxymethyl cellulose (CMC) orally).

The article "Bioactive Fraction of Annona reticulata Bark (or) Ziziphus jujuba Root Bark along with Insulin Attenuates Painful Diabetic Neuropathy through Inhibiting NF-κB Inflammatory Cascade" was published in 2017. Journal: Front Cell Neurosci.

**Group-II:** Animals with diabetes + vehicle treatment (0.3% CMC orally).

**Group-III:** Animals with diabetes + Insulin (5 IU/kg s.c.).

**Group-IV:** Animals with diabetes + Insulin (5 IU/kg s.c.) + Pregabalin (100 mg/kg orally).

**Group-V and VI:** Animals with diabetes + Insulin (5 IU/kg s.c.) + Oral gavage of ARBME (200 mg/kg) and ARBME (400 mg/kg).

**Group-VII and VIII:** Animals with diabetes + Insulin (5 IU/kg s.c.) + Oral gavage of ARBWF (50 mg/kg) and ARBWF (100 mg/kg).

**Group-XI and X:** Animals with diabetes + Insulin (5 IU/kg s.c.) + Oral gavage of ZJME (200 mg/kg) and ZJME (400 mg/kg) respectively.

**Group-XI and XII:** Animals with diabetes + Insulin (5 IU/kg s.c.) + Oral gavage of ZJWF (50 mg/kg) and ZJWF (100 mg/kg) respectively.

**Note:** Plant extracts and fractions were suspended in 0.3% CMC and fed the rats through oral gavage. Insulin injected through subcutaneous route.

Behavioral assessments like thermal and mechanical hyperalgesia were performed on 0th, 4th, 6th, and 8th week of the study. At the end of the 8th week, animals in all the groups were sacrificed by inhalation anesthesia to collect sciatic nerve and stored in liquid nitrogen for biochemical estimation (SOD, CAT, LPO, GSH, IL-1β, IL-6, IL-10, and TNF-α).

### Behavioral assessment

#### Hot plate test (thermal hyperalgesia)

Animals from all the groups were placed individually on Eddy's hot plate (55 ± 1°C). The first sight of paw licking and jumping was considered as escape latency and measured in seconds. To avoid the damage to the animal paw, cut-off time was set to be 10 s (Salat et al., 2014).

#### Tail immersion test (thermal hyperalgesia)

The lower portion of the tail tip (5 cm) was marked and immersed in the hot water (52.5 ± 1°C). The tail withdrawal latency was recorded in seconds and the test was repeated three times with at least 15 min interval. Cut-off time was set to be 15 s (Sharma et al., 2006).

#### Cold plate test (thermal allodynia)

Animals were kept on the ice platform submerged about 1 cm below the surface of the chilled water (4°C), such that glabrous skin of animal feet in contact with the chilled water. The escape latency time was recorded with the cutoff time 30 s (Ranjithkumar et al., 2013).

#### Randall-selitto test (mechanical hyperalgesia)

The nociceptive threshold of the animals was measured following Randall and Selitto procedure. Animals were habituated to the laboratory environment before 1 h of the experiment with water and food being withdrawn. Nociceptive threshold was measured in grams by Randall-Selitto pressure analgesia meter (Panlab Harvard Apparatus, Spain). Pressure on the paw was increasing continuously until the animal was withdrawn the paw. To prevent the damage to the paw, cutoff point was set to be 300 g.

The article "Bioactive Fraction of Annona reticulata Bark (or) Ziziphus jujuba Root Bark along with Insulin Attenuates Painful Diabetic Neuropathy through Inhibiting NF-κB Inflammatory Cascade" was published in 2017. Journal: Front Cell Neurosci.

#### Measurement of % response of various treatments against DNP in all pain models

After 8 weeks of drug treatment period the percentage response of each drug treatment with respective to non-treatment in various pain models (hot plate, tail immersion, cold plate and paw pressure) were calculated by the following formula:

(1) $$\text{Response }=\;\frac{\begin{array}{c} 8\text{th week drug treatment group reading}\\ -8\text{th week vehicle treatment group reading} \end{array}}{8\text{th week vehicle treatment group reading}}\;\times \;100$$

8th week drug treatment group reading: Pain evaluation readings at 8th week of diabetic animals treated with insulin (5 IU/kg), and pregabalin (100 mg/kg), ARBME (200 and 400 mg/kg), ARBWF (50 and 100 mg/kg), ZJME (200 and 400 mg/kg), and ZJWF (50 and 100 mg/kg) treatments along with insulin (5 IU/kg).

8th week vehicle treatment group reading: Pain evaluation readings at 8th week of diabetic animals treated with vehicle (2 ml/kg) alone.

### Estimation of biochemical parameters

#### Tissue collection and lysate preparation

At the end of the 8th week of drug treatment, all the animals were sacrificed and whole sciatic nerve was isolated immediately in liquid nitrogen and carried to laboratory from animal house. Sciatic nerve homogenate (10% w/v) was prepared with 0.1 M Tris-HCl buffer (pH 7.4). Homogenates were centrifuged at 10 K rpm for 15 min (4°C) and the supernatant was collected separately for biochemical estimation (Naik et al., 2006).

#### Determination of antioxidant enzymes and lipid peroxidation

Supernatant was employed to estimate SOD and catalase (CAT), from biochemical kits from Sigma-Aldrich according to the protocol given by the manufacturer. Reduced glutathione (GSH) levels were measured by following Kandimalla et al. (2016c). Lipid peroxidation was determined by measuring the thiobarbituric acid reactive substances (TBARS) (Ohkawa et al., 1979).

#### Determination of cytokine levels

Levels IL-1β, IL-6, IL-10, and TNF-α, were determined by kits available from RandD systems, USA as per the instructions given by the manufacturer (Kandimalla et al., 2016c,d; Kalita et al., 2017).

#### Western blot analysis to measure NF-κB and iNOS expression

Sciatic nerve was homogenized with lysis buffer containing protease inhibitors 1 mg/ml leupeptin, 1 mg/ml aprotinin, 1% Triton X-100, 1 mM EDTA, 150 mM NaCl, 2.5 mM sodium pyrophosphate, 1 mM Na3VO4, 1 mM b-glycerophosphate, and 20 mM Tris (pH 7.5) to obtain the protein lysate. Protein separation was done by SDS-PAGE by loading equal quantity of total protein in each well. Further, protein bands were transferred to nitrocellulose membrane (Cell Signaling, USA). Non-specific proteins were blocked by 5% fat-free milk powder, and membranes were incubated with primary antibody NF-κB and iNOS (1: 1,000) (Cell Signaling Technology, USA) separately for 12 h at 4°C. Membranes were washed with washing buffer and incubated with horseradish peroxidase secondary antibody (1: 20,00). Bands were visualized under Chemidoc system (BioRad, USA) using ECL kit (BioRad, USA). β-actin expression was also measured to confirm the equal loading of the protein.

The article "Bioactive Fraction of Annona reticulata Bark (or) Ziziphus jujuba Root Bark along with Insulin Attenuates Painful Diabetic Neuropathy through Inhibiting NF-κB Inflammatory Cascade" was published in 2017. Journal: Front Cell Neurosci.

#### Statistical analysis

All the results were expressed in mean ± standard deviation. One way ANOVA followed by Bonferroni *post-hoc* test was performed to find the significant difference between the treatment groups. A *p* ≤ 0.05 was considered as significant. All the statistical analysis carried out in this study was done with GraphPad Prism 6 software.

## Results

### Neuroprotective effect of *A. reticulata* and *Z. jujuba* fractions on SHSY5Y cells

We have evaluated the effect of DMSO, H_2_O_2_ and all the plant fractions on the cell viability of SHSY5Y cells. The results showed that DMSO and plant fractions at tested concentrations did not affect the cell viability of SHSY5Y cells. H_2_O_2_ treatment at 100 μM concentration significantly decreases the cell viability to 64% compared to control group. This result indicates that H_2_O_2_ causes potential damage to neuron cells. Bioactive fractions of ARB and ZJ- Hexane (ARBHF and ZJHF), chloroform (ARBCF and ZJCF), ethyl acetate (ARBEAF and ZJEAF) and methanol residue (ARBMR and ZJMR) did not exhibited significant protection from H_2_O_2_ toxicity. Whereas methanol extract (ARBME and ZJME) and its water fraction (ARBWF and ZJWF) showed significant (*p* ≤ 0.05) protection from H_2_O_2_ dose dependently (Table 1). Neuroprotection by these fractions were further confirmed by the LDH and TBARS levels measurement. H_2_O_2_ treatment leads to significant increase in the TBARS levels and LDH leakage from the SHSY5Y cells into the culture media. Whereas cells pretreated with ARBME, ARBWF, ZJME, and ZJWF showed less levels of TBARS and LDH leakage. LDH assay and TBARS results further strengthen the neuroprotective ability of the plant fractions. Among all the fractions tested water fractions (ARBWF and ZJWF) of both the plants were found to be potent than the methanol extracts (ARBME and ZJME). From these *in vitro* results, ARBME, ZJME, ARBWF, and ZJWF were selected for further evaluation using animal models.

**Table 1:** **Protective effect of ***A. reticulata*** and ***Z. jujuba*** plant extracts and fractions against H_**2**_O_**2**_ intoxicated SHSY5Y cell lines**.

**Group no**.	**Treatment**	**Concentration**	**% Cell viability**	**LDH (U/L)**	**TBARS (nmol/mg protein)**
Group-I (Control)	Normal	No treatment	98.5 ± 1.84	84.6 ± 0.94	1.84 ± 0.08
	DMSO	0.25% V/V	97.8 ± 2.12	85.7 ± 1.03	1.87 ± 0.07
	ARBME	200 μg/ml	96.8 ± 1.73	86.2 ± 0.82	1.86 ± 0.07
	ARBHF	200 μg/ml	96.5 ± 1.66	85.4 ± 0.97	1.78 ± 0.08
	ARBCF	200 μg/ml	96.7 ± 2.03	86.6 ± 1.12	1.81 ± 0.07
	ARBEAF	200 μg/ml	96.2 ± 1.85	85.2 ± 1.07	1.89 ± 0.09
	ARBWF	200 μg/ml	96.4 ± 1.92	86.8 ± 0.96	1.86 ± 0.08
	ARBMR	200 μg/ml	96.7 ± 1.64	85.6 ± 0.81	1.82 ± 0.07
	ZJME	200 μg/ml	97.1 ± 2.16	85.2 ± 0.88	1.79 ± 0.08
	ZJHF	200 μg/ml	96.7 ± 1.78	85.6 ± 0.96	1.88 ± 0.09
	ZJCF	200 μg/ml	96.4 ± 1.46	86.1 ± 1.14	1.85 ± 0.08
	ZJEAF	200 μg/ml	97.3 ± 2.07	85.7 ± 0.86	1.87 ± 0.09
	ZJWF	200 μg/ml	96.8 ± 1.62	86.8 ± 0.95	1.83 ± 0.07
	ZJMR	200 μg/ml	96.6 ± 2.15	85.8 ± 1.12	1.78 ± 0.08
Group-II	H_2_O_2_ control	100 μM	38.7 ± 2.73^∧^	157.9 ± 4.26^∧^	4.28 ± 0.24^∧^
Group-III	ARBME + H_2_O_2_	50 μg/ml + 100 μM	69.2 ± 3.47^*^	117.4 ± 3.16^*^	2.97 ± 0.17^*^
		100 μg/ml + 100 μM	76.4 ± 3.82^*^	106.8 ± 2.68^*^	2.53 ± 0.15^*^
		200 μg/ml + 100 μM	84.6 ± 3.25^*^^#^	94.2 ± 2.19^*^^#^	2.18 ± 0.11^*^^#^
	ARBHF + H_2_O_2_	50 μg/ml + 100 μM	41.2 ± 2.81	152.4 ± 3.62	4.12 ± 0.21
		100 μg/ml + 100 μM	43.6 ± 2.64	151.7 ± 3.85	4.06 ± 0.23
		200 μg/ml + 100 μM	43.9 ± 3.54	150.5 ± 4.16	4.04 ± 0.21
	ARBCF + H_2_O_2_	50 μg/ml + 100 μM	39.5 ± 3.17	157.2 ± 4.07	4.15 ± 0.26
		100 μg/ml + 100 μM	40.8 ± 2.62	155.2 ± 3.42	4.11 ± 0.23
		200 μg/ml + 100 μM	41.7 ± 2.86	152.8 ± 4.21	4.08 ± 0.19
	ARBEAF + H_2_O_2_	50 μg/ml + 100 μM	40.4 ± 3.45	156.7 ± 3.27	4.09 ± 0.22
		100 μg/ml + 100 μM	41.8 ± 2.69	153.5 ± 4.11	4.08 ± 0.25
		200 μg/ml + 100 μM	42.6 ± 3.14	152.1 ± 3.68	4.02 ± 0.19
	ARBWF + H_2_O_2_	50 μg/ml + 100 μM	78.6 ± 3.86^*^	104.8 ± 2.59^*^	2.56 ± 0.11^*^
		100 μg/ml + 100 μM	86.2 ± 4.17^*^	90.7 ± 2.81^*^	2.21 ± 0.13^*^
		200 μg/ml + 100 μM	92.1 ± 3.66^*^^#^	88.2 ± 2.44^*^^#^	2.02 ± 0.09^*^^#^
	ARBMR + H_2_O_2_	50 μg/ml + 100 μM	44.5 ± 3.92	142.6 ± 3.27	3.46 ± 0.17
		100 μg/ml + 100 μM	49.8 ± 2.73	137.8 ± 3.41	3.24 ± 0.18
		200 μg/ml + 100 μM	55.3 ± 4.14^*^	131.2 ± 2.85^*^	3.11 ± 0.16^*^
Group-IV	ZJME + H_2_O_2_	50 μg/ml + 100 μM	72.8 ± 4.27^*^	114.3 ± 3.62^*^	2.72 ± 0.19^*^
		100 μg/ml + 100 μM	79.6 ± 3.62^*^	102.6 ± 3.05^*^^#^	2.44 ± 0.14^*^
		200 μg/ml + 100 μM	88.5 ± 4.08^*^^#^	89.7 ± 2.43^*^^#^	2.07 ± 0.12^*^^#^
	ZJHF + H_2_O_2_	50 μg/ml + 100 μM	40.8 ± 3.48	155.2 ± 4.16	4.02 ± 0.19
		100 μg/ml + 100 μM	41.2 ± 2.86	152.8 ± 3.45	3.97 ± 0.21
		200 μg/ml + 100 μM	41.8 ± 3.16	151.9 ± 4.21	3.92 ± 0.18
	ZJCF + H_2_O_2_	50 μg/ml + 100 μM	39.2 ± 2.44	158.2 ± 3.86	4.07 ± 0.23
		100 μg/ml + 100 μM	40.3 ± 3.24	156.4 ± 4.08	4.01 ± 0.17
		200 μg/ml + 100 μM	41.1 ± 2.61	154.3 ± 3.58	3.95 ± 0.19
	ZJEAF + H_2_O_2_	50 μg/ml + 100 μM	43.7 ± 2.54	149.6 ± 2.96	4.03 ± 0.19
		100 μg/ml + 100 μM	44.2 ± 3.16	148.2 ± 3.38	3.94 ± 0.21
		200 μg/ml + 100 μM	44.9 ± 3.32	147.1 ± 3.02	3.88 ± 0.21
	ZJWF + H_2_O_2_	50 μg/ml + 100 μM	80.7 ± 4.38^*^	101.7 ± 2.47^*^	2.41 ± 0.14^*^
		100 μg/ml + 100 μM	89.6 ± 4.72^*^	88.1 ± 2.13^*^^#^	2.08 ± 0.11^*^
		200 μg/ml + 100 μM	94.7 ± 5.16^*^^#^	86.8 ± 2.26^*^^#^	1.91 ± 0.08^*^^#^
	ZJMR + H_2_O_2_	50 μg/ml + 100 μM	42.4 ± 4.11	150.6 ± 3.11	3.73 ± 0.22
		100 μg/ml + 100 μM	43.5 ± 3.78	149.2 ± 2.94	3.59 ± 0.17
		200 μg/ml + 100 μM	44.7 ± 3.21	148.4 ± 3.01	3.45 ± 0.19

*All the results were presented in mean ± S.D (n = 5)*.

∧ *p ≤ 0.05 in comparison of toxin treated control group (Group-II) with normal control*.

* *p ≤ 0.05 in comparison of group-III and IV with group-II*.

The article "Bioactive Fraction of Annona reticulata Bark (or) Ziziphus jujuba Root Bark along with Insulin Attenuates Painful Diabetic Neuropathy through Inhibiting NF-κB Inflammatory Cascade" was published in 2017. Journal: Front Cell Neurosci.

# *p ≤ 0.05 in comparison between the different doses of same treatment. ARBME: A. reticulata bark methanol extract; ARBHF, A. reticulata bark hexane fraction; ARBCF, A. reticulata bark chloroform fraction; ARBEAF, A. reticulata bark ethyl acetate fraction; ARBWF, A. reticulata bark water fraction; ARBMR, A. reticulata bark methanol residue. ZJME, Z. jujuba root bark methanol extract; ZJHF, Z. jujuba root bark hexane fraction; ZJCF, Z. jujuba root bark chloroform fraction; ZJEAF, Z. jujuba root bark ethyl acetate fraction; ZJWF, Z. jujuba root bark water fraction; ZJMR, Z. jujuba root bark methanol residue*.

### Neuroprotective effect of *A. reticulata* and *Z. jujuba* active fractions on DRG neuronal cells

MTT assay results depicted that H_2_O_2_ (100 μM) caused significant (*p* ≤ 0.05) decline in the cell viability of DRG neurons compared to normal control. DMSO (0.1% v/v), ARBME, ARBWF, ZJME, and ZJWF at 200 μg/ml did not showed adverse effect on cell viability. Further DRG cells pre-treated with ARBME, ARBWF, ZJME, and ZJWF showed significant neuroprotection (*p* ≤ 0.05) from H_2_O_2_ in a dose dependent manner compared to H_2_O_2_ alone treated cells (Table 2).

**Table 2:** **Protective effect of ***A. reticulata*** and ***Z. jujuba*** active plant fractions against H_**2**_O_**2**_ intoxicated DRG neuronal cells**.

**Group no**.	**Treatment**	**Concentration**	**% Cell viability**
Group-I (Control)	Normal	No treatment	99.2 ± 3.26
	DMSO	0.1% V/V	98.5 ± 3.78
	ARBME	200 μg/ml	98.7 ± 3.18
	ARBWF	200 μg/ml	98.1 ± 2.94
	ZJME	200 μg/ml	98.3 ± 3.41
	ZJWF	200 μg/ml	97.8 ± 3.08
Group-II	H_2_O_2_ control	100 μM	51.3 ± 4.73^∧^
Group-III	ARBME + H_2_O_2_	50 μg/ml + 100 μM	72.6 ± 5.13^*^
		100 μg/ml + 100 μM	81.8 ± 4.84^*^
		200 μg/ml + 100 μM	87.1 ± 4.63^*^
	ARBWF + H_2_O_2_	50 μg/ml + 100 μM	76.9 ± 4.38^*^
		100 μg/ml + 100 μM	85.2 ± 3.94^*^
		200 μg/ml + 100 μM	89.5 ± 4.46^*^
Group-IV	ZJME + H_2_O_2_	50 μg/ml + 100 μM	74.8 ± 3.88^*^
		100 μg/ml + 100 μM	81.1 ± 5.07^*^
		200 μg/ml + 100 μM	88.6 ± 4.27^*^
	ZJWF + H_2_O_2_	50 μg/ml + 100 μM	79.4 ± 5.16^*^
		100 μg/ml + 100 μM	87.3 ± 4.48^*^
		200 μg/ml + 100 μM	92.5 ± 3.69^*^

*All the results were presented in mean ± S.D (n = 5)*.

∧ *p ≤ 0.05 in comparison of toxin treated control group (Group-II) with normal control*.

* *p ≤ 0.05 in comparison of group-III and IV with group-II. ARBME, A. reticulata bark methanol extract; ARBWF, A. reticulata bark water fraction; ZJME, Z. jujuba root bark methanol extract; ZJWF, Z. jujuba root bark water fraction*.

The article "Bioactive Fraction of Annona reticulata Bark (or) Ziziphus jujuba Root Bark along with Insulin Attenuates Painful Diabetic Neuropathy through Inhibiting NF-κB Inflammatory Cascade" was published in 2017. Journal: Front Cell Neurosci.

### Acute toxicity studies

All the tested fractions (ARBME, ARBWF, ZJME, and ZJWF) at 2,000 mg/kg and same fractions along with insulin (5 IU/kg) did not show any effect on heart rate, respiratory rate, corneal reflex, body temperature, salivation, locomotor activity, skin tone, body tone, abdominal tone, grip strength, tremors, tail elevation, piloerection, twitches, and convulsions. During 14 days of the observation period, no mortality was observed in extract treated animals. Acute toxicity study results conclude that ARBME, ARBWF, ZJME, and ZJWF were non-toxic to the animals at tested concentration. So we further continued the *in vivo* experiments on these plant fractions against diabetic neuropathy.

### Effect of different drug treatment on body weight and fasting blood glucose

Diabetic animals treated with vehicle (2 ml/kg) showed significant (*p* ≤ 0.05) decline in body weight at 8th week compared with sham control group 8th week. Where there was no significant difference in body weight was observed in animals treated pregabalin (100 mg/kg), ARBME (200 and 400 mg/kg), ARBWF (50 and 100 mg/kg), ZJME (200 and 400 mg/kg), ZJWF (50 and 100 mg/kg) treatments along with insulin (5 IU/kg) at 8th week compared with insulin (5 IU/kg) alone treated animals. STZ (50 mg/kg) treatment causes significant (*p* ≤ 0.05) rise in FBG levels of all treatment groups at 1st week. Further, treatment with insulin (5 IU/kg) alone causes a significant (*p* ≤ 0.05) decline in the FBG levels at 8th week compared to diabetic control at 8th week. Further standard drug pregabalin (100 mg/kg), ARBME (200 mg and 400 mg/kg), ARBWF (50 mg/kg), ZJME (200 mg/kg), and ZJWF (50 mg/kg) treatment along with insulin did not decrease the FBG levels significantly compared to insulin alone treated group. However, ZJME at 400 mg/kg, ARBWF and ZJWF at 100 mg/kg treatment along with insulin cause further significant (*p* ≤ 0.05) reduction in FBG levels compared to insulin alone treated animals (Table 3).

The article "Bioactive Fraction of Annona reticulata Bark (or) Ziziphus jujuba Root Bark along with Insulin Attenuates Painful Diabetic Neuropathy through Inhibiting NF-κB Inflammatory Cascade" was published in 2017. Journal: Front Cell Neurosci.

**Table 3:** **Effect of different drug treatment on body weight and blood glucose at different intervals**.

**Group**	**Treatment**	**Body weight (gm)**			**FBG (mg/dl)**		
		**0th week**	**1st week**	**8th week**	**0th week**	**1st week**	**8th week**
I	Normal animals (Sham control)	225.8 ± 8.1	226.2 ± 8.2	229.4 ± 7.9	98.1 ± 8.8	97.8 ± 8.6	98.3 ± 7.2
II	Diabetic control	224.9 ± 7.2	224.5 ± 7.4	194.7 ± 9.2^∧^	96.4 ± 7.5	294.8 ± 17.8	346.2 ± 27.4^∧^
III	Diabetic animals + Insulin (5 IU/kg)	222.5 ± 8.4	221.8 ± 8.6	217.5 ± 7.9	101.2 ± 6.9	284.5 ± 21.6	132.7 ± 14.8^*^
IV	Diabetic animals+ Pregabalin (100 mg/kg)+ Insulin (5 IU/kg)	226.2 ± 9.4	225.7 ± 9.6	219.2 ± 7.5	98.7 ± 6.8	289.4 ± 24.8	137.2 ± 16.4^*^
V	Diabetic animals+ ARBME (200 mg/kg)+ Insulin (5 IU/kg)	223.8 ± 6.6	223.2 ± 6.8	216.8 ± 8.4	100.6 ± 7.4	275.9 ± 18.4	126.5 ± 14.3^*^
VI	Diabetic animals+ ARBME (400 mg/kg)+ Insulin (5 IU/kg)	226.3 ± 7.9	225.7 ± 8.1	214.8 ± 9.3	97.5 ± 6.7	296.7 ± 22.4	115.8 ± 13.6^*^
VII	Diabetic animals+ ARBWF (50 mg/kg) Insulin+ (5 IU/kg)	223.4 ± 7.8	222.8 ± 7.6	214.3 ± 6.2	101.8 ± 8.2	272.6 ± 26.1	122.9 ± 14.3^*^
VIII	Diabetic animals+ ARBWF (100 mg/kg)+ Insulin (5 IU/kg)	226.9 ± 9.9	226.5 ± 10.3	217.6 ± 7.7	98.6 ± 7.3	294.3 ± 18.3	107.5 ± 10.9^*^^$^
IX	Diabetic animals+ ZJME (200 mg/kg)+ Insulin (5 IU/kg)	226.3 ± 8.5	225.9 ± 8.3	215.2 ± 8.6	99.4 ± 8.4	277.4 ± 20.6	131.2 ± 14.6^*^
X	Diabetic animals+ ZJME (400 mg/kg)+ Insulin (5 IU/kg)	224.1 ± 9.3	223.6 ± 9.5	214.7 ± 6.8	101.2 ± 8.1	295.2 ± 16.8	109.6 ± 13.7^*^^$^^#^
XI	Diabetic animals+ ZJWF (50 mg/kg)+ Insulin (5 IU/kg)	224.9 ± 10.2	224.3 ± 10.6	217.8 ± 7.9	97.7 ± 7.5	276.1 ± 27.5	124.8 ± 16.3^*^
XII	Diabetic animals+ ZJWF (100 mg/kg)+ Insulin (5 IU/kg)	226.6 ± 9.6	226.3 ± 9.8	216.4 ± 10.2	96.5 ± 7.2	284.9 ± 21.4	103.6 ± 12.8^*^^$^^#^

*All the results were presented in mean ± S.D (n = 6)*.

∧ *p ≤ 0.05 in comparison of diabetic animals (Group-II) with normal animals (Group-I)*.

* *p ≤ 0.05 in comparison of drug treated groups (Group: III–XII) with diabetic control group (Group: II)*.

$ *p ≤ 0.05 in comparison of drug treatment along with insulin treated groups (Group: IV–XII) with insulin alone treated group (Group-III)*.

# *p ≤ 0.05 in comparison between the different doses of same treatment groups. ARBME, A. reticulata bark methanol extract; ARBWF, A. reticulata bark water fraction; ZJME, Z. jujuba root bark methanol extract; ZJWF, Z. jujuba root bark water fraction*.

### Effect of different drug treatment on behavioral parameters

#### Thermal hyperalgesia (hot plate and tail immersion tests)

A significant decrease (*p* ≤ 0.05) in the escape latency period was observed at 4th week in diabetes induced animals compared to the 0th week. This decrease was consistent up to 8th week in vehicle (2 ml/kg) alone treated animals. Where as in sham control group there was no significant difference in the escape latency period was observed. Insulin (5 IU/kg) treatment alone fails to improve this condition as no significant difference in escape latency period was observed at 6th and 8th week compared with 4th week. Further pregabalin (100 mg/kg), ARBME (200 and 400 mg/kg), ARBWF (50 and 100 mg/kg), ZJME (200 and 400 mg/kg), and ZJWF (50 and 100 mg/kg) along with insulin (5 IU/kg) decreases the thermal hyperalgesia, where a significant (*p* ≤ 0.05) increase in escape latency period was observed at 6th and 8th week of treatment compared with 4th week. We also observed a significant increase in escape latency period at 6th and 8th week compared with 6th and 8th week escape latency period of insulin alone treated animals respectively (Figures 2, 3).

The article "Bioactive Fraction of Annona reticulata Bark (or) Ziziphus jujuba Root Bark along with Insulin Attenuates Painful Diabetic Neuropathy through Inhibiting NF-κB Inflammatory Cascade" was published in 2017. Journal: Front Cell Neurosci.

**Figure 2:** **Effect of different drug treatment on thermal hyperalgesia induced by hot plate method in diabetic neuropathic animals at different time intervals**. All the results were expressed in mean ± S.D (*n* = 6). ^∧^ is *p* ≤ 0.05 in comparison of 4th week with 0th week. ^*^ is *p* ≤ 0.05 in comparison of 6th and 8th week with 4th week. $ is *p* ≤ 0.05 in comparison with insulin alone treated diabetic group at corresponding weeks. ARBME, *A*. *reticulata* bark methanol extract; ARBWF, *A*. *reticulata* bark water fraction; ZJME, *Z. jujuba* root bark methanol extract; ZJWF, *Z*. *jujuba* root bark water fraction.

**Figure 3:** **Effect of different drug treatment on thermal hyperalgesia induced by tail immersion method in diabetic neuropathic animals at different time intervals**. All the results were expressed in mean ± S.D (*n* = 6). ^∧^ is *p* ≤ 0.05 in comparison of 4th week with 0th week. ^*^ is *p* ≤ 0.05 in comparison of 6th and 8th week with 4th week. $ is *p* ≤ 0.05 in comparison with insulin alone treated diabetic group at corresponding weeks. ARBME, *A*. *reticulata* bark methanol extract; ARBWF, *A*. *reticulata* bark water fraction; ZJME, *Z*. *jujuba* root bark methanol extract; ZJWF, *Z*. *jujuba* root bark water fraction.

#### Thermal allodynia (cold plate test)

Diabetes induced animals showed significant (*p* ≤ 0.05) decrease in escape latency period at 4th week compared to 0th week response; this decline was maintained until the end of the study (8th week) in vehicle alone treated animals. Whereas in sham control group there was no significant changes observed throughout the study. Pregabalin (100 mg/kg), ARBME (200 and 400 mg/kg), ARBWF (50 and 100 mg/kg), ZJME (200 and 400 mg/kg), and ZJWF (50 and 100 mg/kg) treatments along with insulin (5 IU/kg) cause significant increase (*p* ≤ 0.05) in escape latency period at 6th and 8th week compared to 4th week response. In this study even insulin (5 IU/kg) treatment alone causes reversal of cold allodynia at 6th and 8th week significantly (*p* ≤ 0.05) compared with 4th week (Figure 4). In this test ARBME, ZJME, ARBWF, and ZJWF at tested high dose resulted in complete reversal of allodynia.

The article "Bioactive Fraction of Annona reticulata Bark (or) Ziziphus jujuba Root Bark along with Insulin Attenuates Painful Diabetic Neuropathy through Inhibiting NF-κB Inflammatory Cascade" was published in 2017. Journal: Front Cell Neurosci.

**Figure 4:** **Effect of different drug treatment on thermal allodynia induced by cold plate method in diabetic neuropathic animals at different time intervals**. All the results were expressed in mean ± S.D (*n* = 6). ^∧^ is *p* ≤ 0.05 in comparison of 4th week with 0th week. ^*^ is *p* ≤ 0.05 in comparison of 6th and 8th week with 4th week. $ is *p* ≤ 0.05 in comparison with insulin alone treated diabetic group at corresponding weeks. ARBME, *A*. *reticulata* bark methanol extract; ARBWF, *A*. *reticulata* bark water fraction; ZJME, *Z*. *jujuba* root bark methanol extract; ZJWF, *Z*. *jujuba* root bark water fraction.

#### Mechanical hyperalgesia (randall-selitto test)

Results of mechanical hyperalgesia reveals that diabetic animals produce significant (*p* ≤ 0.05) decrease in paw withdrawal threshold at 4th week compared to 0th week basal value. Consistent declaim was observed in vehicle alone treated animals. No significant difference was observed at different weeks in animals of sham control group. Insulin (5 IU/kg) alone treated diabetic animals were showed no recovery from this condition at 6th and 8th week of treatment. However, Pregabalin (100 mg/kg), ARBME (200 and 400 mg/kg), ARBWF (50 and 100 mg/kg), ZJME (200 and 400 mg/kg), and ZJWF (50 and 100 mg/kg) treatments along with insulin (5 IU/kg) potentially increase the paw withdrawal threshold at 6th and 8th week compared to 4th week. We have further observed a significant (*p* ≤ 0.05) increase in paw withdrawal threshold at 6th and 8th week compared with 6th and 8th week paw withdrawal threshold of insulin alone treated animals respectively (Figure 5).

**Figure 5:** **Effect of different drug treatment on mechanical hyperalgesia induced by paw pressure analgesiometer method in diabetic neuropathic animals at different time intervals**. All the results were expressed in mean ± S.D (*n* = 6). ^∧^ is *p* ≤ 0.05 in comparison of 4th week with 0th week. ^*^ is *p* ≤ 0.05 in comparison of 6th and 8th week with 4th week. $ is *p* ≤ 0.05 in comparison with insulin alone treated diabetic group at corresponding weeks. ARBME, *A*. *reticulata* bark methanol extract; ARBWF, *A*. *reticulata* bark water fraction; ZJME, *Z*. *jujuba* root bark methanol extract; ZJWF, *Z*. *jujuba* root bark water fraction.

The article "Bioactive Fraction of Annona reticulata Bark (or) Ziziphus jujuba Root Bark along with Insulin Attenuates Painful Diabetic Neuropathy through Inhibiting NF-κB Inflammatory Cascade" was published in 2017. Journal: Front Cell Neurosci.

#### % response of various treatments against DNP in all pain models

Figure 6 represents the % response of various drug treatments in different pain models of DNP. Animals treated with pregabalin (100 mg/kg), ARBME (200 and 400 mg/kg), ARBWF (50 and 100 mg/kg), ZJME (200 and 400 mg/kg), and ZJWF (50 and 100 mg/kg) along with insulin (5 IU/kg) showed significant (*p* ≤ 0.05) increase in the % response compared to insulin (5 IU/kg) alone treated animals in hot plate, tail immersion and Randall-Selitto tests. But in cold plate measurement; only ZJME (400 mg/kg), ARBWF (100 mg/kg), and ZJWF (100 mg/kg) along with insulin (5 IU/kg), showed significant difference in % response compared to insulin (5 IU/kg) alone treatment group.

**Figure 6:** **Effect of different drug treatments on % response in various pain models**. (A) Insulin (5 IU/kg); (B) Pregabalin (100 mg/kg) + Insulin (5 IU/kg); (C) ARBME (200 mg/kg) + Insulin (5 IU/kg); (D) ARBME (400 mg/kg) + Insulin (5 IU/kg); (E) ARBWF (50 mg/kg) + Insulin (5 IU/kg); (F) ARBWF (100 mg/kg) + Insulin (5 IU/kg); (G) ZJME (200 mg/kg) + Insulin (5 IU/kg); (H) ZJME (400 mg/kg) + Insulin (5 IU/kg); (I) ZJWF (50 mg/kg) + Insulin (5 IU/kg); (J) ZJWF (100 mg/kg) + Insulin (5 IU/kg). All the results were expressed in mean ± S.D. ^*^ is *p* ≤ 0.05 in comparison of (B–J) with (A).

#### Effect of drug treatment on lipid peroxidation

A significant (*p* ≤ 0.05) increase in the LPO was observed in diabetic animals compared to non-diabetic animals (Sham control). Insulin (5 IU/kg) along with pregabalin (100 mg/kg), ARBME (200 and 400 mg/kg), ARBWF (50 and 100 mg/kg), ZJME (200 and 400 mg/kg), and ZJWF (50 and 100 mg/kg) treatment significantly (*p* ≤ 0.05) decrease d the LPO levels compared to diabetic animals. Where insulin (5 IU/kg) treatment alone fails to significantly lowering down the LPO levels than diabetic control. Further, except pregabalin (100 mg/kg), ARBME (200 mg/kg) along with Insulin (5 IU/kg) all the other drug treatment groups showed significantly (*p* ≤ 0.05) less levels of LPO compared to insulin (5 IU/kg) alone treated animals. ARBWF and ZJWF at both the doses showed strong response than ARBME and ZJME (Table 4).

**Table 4:** **Effect of drug treatment on sciatic nerve lipid peroxidation and antioxidant enzyme levels**.

**Group No**.	**Group**	**SOD (U/ml)**	**CAT (nmol/min/ml)**	**GSH (nm/mg protein)**	**TBARS (nmol/g tissue)**
I	Normal animal (Sham control)	11.8 ± 1.9	6.8 ± 0.7	9.7 ± 0.92	143.8 ± 7.4
II	Diabetic control	3.2 ± 0.9	1.8 ± 0.4^∧^	2.4 ± 0.47^∧^	317.6 ± 14.8^∧^
III	Diabetic animals + Insulin (5 IU/kg)	5.1 ± 1.2^*^	3.2 ± 0.6	4.2 ± 0.64^*^	266.4 ± 16.3
IV	Diabetic animals+ Pregabalin (100 mg/kg)+ Insulin (5 IU/kg)	7.6 ± 1.7^*^^$^	3.9 ± 1.1^*^	5.9 ± 0.75^*^^$^	248.7 ± 13.4^*^
V	Diabetic animals+ ARBME (200 mg/kg)+ Insulin (5 IU/kg)	6.3 ± 1.1^*^	4.1 ± 0.8^*^	5.1 ± 0.68^*^	241.5 ± 12.7^*^
VI	Diabetic animals+ ARBME (400 mg/kg)+ Insulin (5 IU/kg)	7.7 ± 1.4^*^^$^	4.6 ± 0.7^*^	6.5 ± 0.73^*^^$^	219.6 ± 14.6^*^^$^^#^
VII	Diabetic animals+ ARBWF (50 mg/kg) Insulin+ (5 IU/kg)	7.1 ± 1.7^*^	4.4 ± 0.9^*^	6.2 ± 0.59^*^^$^	227.5 ± 15.2^*^^$^
VIII	Diabetic animals+ ARBWF (100 mg/kg)+ Insulin (5 IU/kg)	8.4 ± 1.5^*^^$^	5.1 ± 1.1^*^^$^	7.1 ± 0.84^*^^$^	204.9 ± 12.3^*^^$^
IX	Diabetic animals+ ZJME (200 mg/kg)+ Insulin (5 IU/kg)	6.5 ± 1.6^*^	4.3 ± 0.8^*^	5.3 ± 0.64^*^	233.1 ± 16.8^*^^$^
X	Diabetic animals+ ZJME (400 mg/kg)+ Insulin (5 IU/kg)	7.9 ± 1.8^*^^$^	4.8 ± 0.9^*^	6.9 ± 0.77^*^^$^^#^	211.6 ± 14.4^*^^$^^#^
XI	Diabetic animals+ ZJWF (50 mg/kg)+ Insulin (5 IU/kg)	7.4 ± 1.4^*^^$^	4.7 ± 1.3^*^	6.5 ± 0.71^*^^$^	220.4 ± 12.3^*^^$^
XII	Diabetic animals+ ZJWF (100 mg/kg)+ Insulin (5 IU/kg)	8.7 ± 1.7^*^^$^	5.4 ± 1.2^*^^$^	7.6 ± 0.87^*^^$^	196.2 ± 16.6^*^^$^^#^

*All the results were presented in mean ± S.D (n = 6)*.

∧ *p ≤ 0.05 in comparison of diabetic animals (Group-II) with normal animals (Group-I)*.

* *p ≤ 0.05 in comparison of drug treated groups (Group-III–XII) with diabetic control group (Group-II)*.

$ *p ≤ 0.05 in comparison of drug treatment along with insulin treated groups (Group-IV to XII) with insulin alone treated group (Group-III)*.

The article "Bioactive Fraction of Annona reticulata Bark (or) Ziziphus jujuba Root Bark along with Insulin Attenuates Painful Diabetic Neuropathy through Inhibiting NF-κB Inflammatory Cascade" was published in 2017. Journal: Front Cell Neurosci.

# *p ≤ 0.05 in comparison between the different doses of same treatment. ARBME, A. reticulata bark methanol extract; ARBWF, A. reticulata bark water fraction; ZJME, Z. jujuba root bark methanol extract; ZJWF, Z. jujuba root bark water fraction*.

#### Effect of drug treatment on antioxidant enzyme levels

Diabetic animals showed a significant (*p* ≤ 0.05) decrease in antioxidant enzymes SOD, CAT and GSH compared to normal animals. A significant (*p* ≤ 0.05) increase in all the tested antioxidant enzymes (SOD, CAT and GSH) was observed in diabetic animals treated with ARBME (200 and 400 mg/kg), ZJME (200 and 400 mg/kg), ARBWF (50 and 100 mg/kg), ZJWF (50 and 100 mg/kg), and pregabalin (100 mg/kg) treatment along with insulin (5 IU/kg) compared to vehicle treated diabetic animals. Insulin (5 IU/kg) alone treated animals also showed a significant (*p* ≤ 0.05) rise in SOD and GSH levels but not CAT when compared to vehicle treated diabetic animals. Further, treatment with pregabalin (100 mg/kg), ARBME (400 mg/kg), ARBWF (100 mg/kg), ZJME (400 mg/kg), ZJWF (50 and 100 mg/kg) along with insulin (5 IU/kg) showed significant (*p* ≤ 0.05) increase in SOD levels compared to insulin (5 IU/kg) alone treated diabetic animals. In case of CAT levels, apart from ARBWF and ZJWF at 100 mg/kg along with insulin (5 IU/kg) no other treatment groups showed significant difference compared to insulin (5 IU/kg) alone treated diabetic animals. Insulin (5 IU/kg) treatment along with ARBME and ZJME at 200 mg/kg did not alter the GSH levels significantly compared to insulin (5 IU/kg) alone treated animals whereas, all the other drug treatments increased significantly (Table 4).

The article "Bioactive Fraction of Annona reticulata Bark (or) Ziziphus jujuba Root Bark along with Insulin Attenuates Painful Diabetic Neuropathy through Inhibiting NF-κB Inflammatory Cascade" was published in 2017. Journal: Front Cell Neurosci.

#### Effect of drug treatment on cytokine levels

At the end of the study, animals from all the treatment groups were measured for cytokine levels. Animals in diabetic control showed significant (*p* ≤ 0.05) increase in all the inflammatory cytokines (IL-1β, IL-6, and TNF-α) and decrease in anti-inflammatory cytokine (IL-10) compared to non-diabetic animals (Sham control). Insulin (5 IU/kg) treatment alone failed to improve this condition. Whereas, pregabalin (100 mg/kg), ARBME (200 and 400 mg/kg), ARBWF (50 and 100 mg/kg), ZJME (200 and 400 mg/kg), and ZJWF (50 and 100 mg/kg) treatment along with insulin (5 IU/kg) showed significant (*p* ≤ 0.05) improvement in impaired levels of all the cytokines compared to diabetic control and insulin (5 IU/kg) alone treated diabetic animals. But, ARBME (200 mg/kg) and ZJME (200 mg/kg) along with insulin (5 IU/kg) did not alter the TNF-α levels further compared to insulin (5 IU/kg) alone treated animals (Figures 7A–D).

**Figure 7:** **Effect of different drug treatment on sciatic nerve (A)** Interleukin-1β **(B)** Interleukin-6 **(C)** tumor necrosis factor-α and **(D)** Interleukin-10 levels in diabetic neuropathic animals. All the results were expressed in mean ± S.D (*n* = 6). ^∧^ is *p* ≤ 0.05 in comparison with normal animals. ^*^ is *p* ≤ 0.05 in comparison with vehicle treated diabetic animals. $ is *p* ≤ 0.05 in comparison with insulin alone treated diabetic group. ARBME, *A*. *reticulata* bark methanol extract; ARBWF, *A*. *reticulata* bark water fraction; ZJME, *Z*. *jujuba* root bark methanol extract; ZJWF, *Z*. *jujuba* root bark water fraction.

#### Effect of drug treatment on NF-κB and iNOS protein expression

Increased expression of inflammatory cytokines is mediated by NF-κB in diabetic neuropathic rats. So, in this present study we measured the effect of plant fractions on NF-κB and iNOS protein levels through western blotting analysis. The blot results reveal that treatment with pregabalin (100 mg/kg), ARBME (400 mg/kg), ZJME (400 mg/kg), ARBWF (100 mg/kg), and ZJWF (100 mg/kg) along with insulin (5 IU/kg) inhibits the NF-κB and iNOS expression compared to diabetic animals. Insulin (5 IU/kg) alone treated animals exhibited no difference in these protein expression levels. Figure 8 explains the NF-κB and iNOS expression in sciatic nerve of the animal from different treatment groups. ARBWF and ZJWF at 100 mg/kg along with insulin (5 IU/kg) treated animals showed better response than animals treated with ARBME and ZJME at 400 mg/kg along with insulin (5 IU/kg). This result demonstrates that polar chemical constituents of methanol extracts of *A. reticulata* bark and *Z. jujuba* root bark play a significant role in controlling inflammation mediated DNP.

The article "Bioactive Fraction of Annona reticulata Bark (or) Ziziphus jujuba Root Bark along with Insulin Attenuates Painful Diabetic Neuropathy through Inhibiting NF-κB Inflammatory Cascade" was published in 2017. Journal: Front Cell Neurosci.

**Figure 8:** **Effect of four week drug treatment on change in expression of NF-κB and iNOS measured by western blotting analysis**. Equal loading was confirmed by β-Actin expression. (1) Normal control (2) Diabetic animals with no treatment; (3) Diabetic animals treated with Insulin (5 IU/kg); (4) Diabetic animals treated with pregabalin (100 mg/kg) + Insulin (5 IU/kg); (5) Diabetic animals treated with ARBME (400 mg/kg) + Insulin (5 IU/kg); (6) Diabetic animals treated with ARBWF (100 mg/kg) + Insulin (5 IU/kg); (7) Diabetic animals treated with ZJME (400 mg/kg) + Insulin (5 IU/kg); (8) Diabetic animals treated with ZJWF (100 mg/kg) + Insulin (5 IU/kg).

## Discussion

In this present study, we evaluated neuroprotective effect of bioactive guided fractions of *A. reticulata* bark and *Z. jujuba* root bark against DNP. The neuroprotective ability of the different plant fractions were tested against SHSY5Y neuroblastoma cell lines. Among all the fractions tested ARBME, ARWF, ZJME, and ZJWF showed neuroprotection against H_2_O_2_ induced death of SHSY5Y cells. The results of MTT assay revealed that H_2_O_2_ treatment cause significant decline in viability of SHSY5Y cells. ARBME, ARWF, ZJME, and ZJWF at tested doses attenuated the toxicity induced by H_2_O_2_ where a significant increase in cell viability was observed in a dose-dependent manner. H_2_O_2_ induced toxicity in SHSY5Y cells is a widely used model to measure the neuroprotective ability of the drugs/pharmaceuticals. H_2_O_2_ is a major ROS that penetrates into the cells and produces highly reactive hydroxyl radicals which involve in the induction of oxidative damage to cell organelles including DNA, lipids, and proteins. This damage leads to the decrease in the viability of the cells (Nirmaladevi et al., 2014). H_2_O_2_ promotes LPO which intern damages the cell membrane with subsequent LDH leakage and necrosis (Garcimartin et al., 2014). LDH is a cytoplasmic enzyme that found in almost all cells of the body. Leakage of the cytosolic enzymes is considered as indication of oxidative stress induced cell damage. H_2_O_2_ treatment caused a significant increase in LPO and LDH leakage from SHSY5Y cell into the culture media which is an indication of oxidative stress mediated cell damage. SHSY5Y cell treated with ARBME, ARWF, ZJME, and ZJWF exhibited neuroprotection against H_2_O_2_ induced damage, which was confirmed by increased cell viability, reduced LPO and LDH leakage. This action was due to the neutralization of peroxide radicles and decrease in membrane lipid peroxidation. These active fractions could be translationable neuroprotective agents which will help to prevent cell death under vulnerability conditions related to excessive ROS production.

The article "Bioactive Fraction of Annona reticulata Bark (or) Ziziphus jujuba Root Bark along with Insulin Attenuates Painful Diabetic Neuropathy through Inhibiting NF-κB Inflammatory Cascade" was published in 2017. Journal: Front Cell Neurosci.

Relay of sensory information to the central nervous system occurs through axons of DRG neurons. They are an experimental target of diabetic neuropathy due to their exuberant metabolism and sensitivity to high glycaemia. Even short term hyperglycemic condition leads to DRG neurons oxidative damage and apoptosis. In painful neuropathy inflammatory factors plays a crucial role in DRG neuronal damage. Therefore, stabilizing oxidative stress and inhibition of inflammation has been considered as mainstream strategies for the treatment of DNP. As discussed above H_2_O_2_ initiate oxidative damage to neuronal cells and leads to cell death. In this study H_2_O_2_ produced significant decline in cell viability of DRG neuronal cells. Due to strong antioxidant ability; ARBME, ARWF, ZJME, and ZJWF demonstrated significant neuroprotection toward H_2_O_2_ induced neuronal damage in DRG cells. From the *in vitro* results, active plant fractions (ARBME, ARWF, ZJME, and ZJWF) were selected to continue the *in vivo* experiment.

STZ induced diabetic model is widely used to precipitate DNP condition (He et al., 2016). In this present study, STZ induced rats showed a significant increase in the FBG levels and decreased nociceptive threshold. Pregabalin has been used as a standard drug in this study which is a selective α2δ subunit of voltage-gated calcium channels antagonist which is an anticonvulsant drug can potentially inhibits the diabetic neuropathy. Diabetic animals treated with pregabalin, ARBME, ARWF, ZJME, and ZJWF along with insulin increased the nociceptive threshold, inhibited the oxidative stress and inflammatory markers. Animals responded to the hot plate test through paw licking and jumping, which mediated through activation of supraspinal sensitive fibers type I and II (Lopes et al., 2009). Endogenous release of tachykinin neuropeptide substance P in the spinal cord involves in the tail withdrawal due to thermal stimuli in tail immersion test (Yashpal et al., 1993). Randall-Selitto test explains the mechanical hyperalgesia response of the animals and the mechanism behind this action is unclear (Srebro et al., 2015). ARBME, ARWF, ZJME, and ZJWF along with insulin produce an antinociceptive effect in diabetic animals with the neuropathic condition in the hot plate, tail immersion, and paw pressure models, which explain that all the plant fractions act through central mechanisms. This antinociceptive response showed by the plant fractions was due to inhibition of the oxidative stress and inflammatory markers. *A. reticulata* and *Z. jujuba* different plant parts have been reported previously for antinociceptive and antiinflammatory activity (Mahajan and Chopda, 2009; Jamkhande et al., 2016). In DN condition, cold allodynia precipitate due to loss of Aδ fibers which lead to sensitization of cold receptors (Ranjithkumar et al., 2013). Reports suggest that degeneration of the nerve fibers occurs due to hyperglycemia mediated ischemia (Nukada, 2014). In this study insulin treatment alone showed reduction in cold allodynia condition which might be linked to the reduction of hyperglycemia. Similar results were reported by the previous studies (Finnerup and Jensen, 2006; Casey et al., 2010; Ranjithkumar et al., 2013). Supplement of pregabalin (100 mg/kg), ARWF and ZJWF (100 mg/kg) along with insulin further significantly decrease the allodynia condition. Results of cold allodynia test reveal that polar chemical constitutes of ARB and ZJ have the ability to treat this condition potentially.

The article "Bioactive Fraction of Annona reticulata Bark (or) Ziziphus jujuba Root Bark along with Insulin Attenuates Painful Diabetic Neuropathy through Inhibiting NF-κB Inflammatory Cascade" was published in 2017. Journal: Front Cell Neurosci.

Hyperglycemia leads to microvascular and macrovascular complications in the diabetic patients through four major pathways–polyol pathway, activation of advanced glycation end products (AGEs), activation of hexosamine pathway and activation of protein kinase C (PKC). Activated AGEs cause receptor mediated oxidative stress and stimulate NF-κB protein complex (Brownlee, 2001) which is capable of activates an inflammatory response. Activation of this protein induces the expression of iNOS, another essential enzyme in the inflammatory process which binds to COX-2 and enhances its activity through S-nitrosylation. Further, nerve damage causes the activation of glial cells and releases the inflammatory neuropoietic cytokines like TNF-α, IL-1β, and IL-6. These pro inflammatory cytokines plays a major role in the development of neuropathic pain in diabetic animals through neuronal degeneration by p38 phosphorylation (Kim et al., 2005; Verri et al., 2006; Cameron and Cotter, 2008; Edwards et al., 2008; Kumar et al., 2012; Chanchal et al., 2016). In DN conditions, mainly sciatic, femoral and peroneal nerves are affected (Deli et al., 2014). Among all these major nerves, sciatic nerve that originates from the spinal cord (L4-L6) (Schmalbruch, 1986) is mainly affected in rats and responsible for pain. Diabetes potentially affects all the spinal cord glial cells which were reported in STZ induced diabetic rats. This activated microglia up regulates the sodium channels and cause sensory changes in dorsal root ganglia (DRG) (Schreiber et al., 2015). Apart from proinflammatory cytokines, antiinflammatory cytokine IL-10 play a crucial role in pathogenesis of DNP. Nerve injury causes the significant reduction of IL-10 in DNP patients which is a potential marker of the disease (Lees et al., 2013). In this study, DN animals with no drug treatment showed significantly lower levels of IL-10. ARBME, ARWF, ZJME, and ZJWF treatment potentially inhibited NF-κB, iNOS expression and related proinflammatory cytokines in sciatic nerve of DN rats and showed increase levels of IL-10. Reduction of this inflammatory cascade in the sciatic nerve might aid in reducing the inflammatory damage in neurons of diabetic animals. Earlier reports suggest that strict hyperglycemic control fails to inhibit the neuropathic condition. This condition might be due to the release of the early neuropoietic cytokines like TNF-α, IL-1β, and IL-6 at the interphase of hyperglycemia induced biochemical changes and nerve damage. In this study insulin treatment alone fails to control the inflammatory markers and related pain in animals (Skundric and Lisak, 2003), whereas supplement of ARBME, ARWF, ZJME, and ZJWF along with insulin inhibit the same. The results of inflammatory cytokines reveal that ARBME, ARWF, ZJME, and ZJWF act peripherally to reduce the DNP.

The article "Bioactive Fraction of Annona reticulata Bark (or) Ziziphus jujuba Root Bark along with Insulin Attenuates Painful Diabetic Neuropathy through Inhibiting NF-κB Inflammatory Cascade" was published in 2017. Journal: Front Cell Neurosci.

ROS generation and related oxidative stress are other major factors in the development of the neuropathic condition in diabetic animals. In the hyperglycemic state, autoxidation of monosaccharides leads to production of severe oxidative stress. Superoxide and hydroxyl radicles mainly cause vascular impairment and endoneurial hypoxia through oxidative damage. Antioxidant enzymes (SOD, CAT, and GSH) provide defense against these oxidative markers which plays an important role in cytoprotection. Nerve cells are penurious in these antioxidant enzymes (Naik et al., 2006) that neutralizes the ROS produced in DN condition. Overproduction of ROS causes total utilization of these antioxidant enzymes in the nerve tissue. These reduced levels of antioxidant enzymes in DN state can act as a marker for oxidative damage. Previous reports also stated that sciatic nerve of DN animals contains significantly lower levels of SOD, CAT, and GSH (Aziza et al., 2014; Ozyigit et al., 2015). Plant phytochemicals can neutralize the ROS and reduces the burden on antioxidant enzymes in neutralizing the same. So, supplement of plant fractions reduces the ROS in DN animals, resulted in the restoration of antioxidant enzymes to normal levels. Further in DN condition, significant increase in LPO was observed which relates to the overproduction of ROS and reduced levels of antioxidant enzymes. All these factors collectively lead to the impairment of neuronal functions (Bonnefont-Rousselot, 2002; Pop-Busui et al., 2002). In this study, diabetic animals treated with ARBME, ARWF, ZJME, and ZJWF along with insulin neutralizes the ROS and provided the protection against oxidative damage and inflammation to sciatic nerve cells. We also hypothesized that treatment with the plant fractions also protects all the other major nerves from oxidative damage that affected in DNP condition. Previous reports on antioxidant and anti-inflammatory potential *A. reticulata* and *Z. jujuba* further strengthen the present study (Chavan et al., 2012a,b; Kandimalla et al., 2016a,e). Where, both plant bioactive fraction shows protection against DNP through reducing oxidative stress and inflammatory cytokines.

The article "Bioactive Fraction of Annona reticulata Bark (or) Ziziphus jujuba Root Bark along with Insulin Attenuates Painful Diabetic Neuropathy through Inhibiting NF-κB Inflammatory Cascade" was published in 2017. Journal: Front Cell Neurosci.

ARBWF and ZJWF showed strong response than ARBME and ZJME in reducing the diabetic neuropathy in all the tests conducted. We hypothesized that strong antioxidant ability of both ARBWF and ZJWF neutralizes the harmful ROS and prevent the lesions of pancreatic beta cells. Where, both the fractions at higher dose further decrease the blood glucose levels compare to insulin treatment alone (Hosseini et al., 2015). Further, both the plant fractions showed significant protection toward nerve fiber from oxidative damage and reduced the pain sensation. The results were comparable with standard drug pregabalin which was reported to have analgesic, anti-inflammatory, anxiolytic and antioxidant property. Pregabalin also have anti-hyperalgesic and anti-allodynia activity in animals with neuropathic pain (Aswar et al., 2014). In this study, pregabalin treatment along with insulin cause significant protection from DNP through inhibiting oxidative stress and inflammatory cytokines. Schematic representation of mechanism of action of active plant fractions was given in Figure 9. The present study explains that chemical constituents of *A. reticulata* and *Z. jujuba* attenuate the DNP through acting both centrally (pain reduction in animal models) and peripherally (reduction of oxidative stress and inflammatory protein markers). Biomarker isolation from both the plants are undergoing at drug discovery laboratory, IASST, Guwahati-35, Assam, India.

The article "Bioactive Fraction of Annona reticulata Bark (or) Ziziphus jujuba Root Bark along with Insulin Attenuates Painful Diabetic Neuropathy through Inhibiting NF-κB Inflammatory Cascade" was published in 2017. Journal: Front Cell Neurosci.

**Figure 9:** **Schematic representation of possible mechanism of action of active plant fractions of ***Annona reticulata*** bark and ***Ziziphus jujuba*** root bark against painful diabetic neuropathy**. ARBME, *A*. *reticulata* bark methanol extract; ARBWF, *A*. *reticulata* bark water fraction; ZJME, *Z*. *jujuba* root bark methanol extract; ZJWF, *Z*. *jujuba* root bark water fraction.

## Author contributions

RK designed the whole study and performed both *in vitro* and *in vivo* experiments. SK helped RK in all the tests conducted. BC helped in cell line experiments. SM helped toward manuscript correction and literature review. RD helped in the literature review. MR and NCT contributed toward study design. JK and SD compiled the results, supervise the experiments and corrected manuscript.

### Conflict of interest statement

A portion of work mentioned in this article was used to file an Indian patent application (No: 201631008543) dated 11th March 2016. The authors declare that the research was conducted in the absence of any commercial or financial relationships that could be construed as a potential conflict of interest.
